The article "Clinical Features and Biomarkers for Early Prediction of Refractory Mycoplasma Pneumoniae Pneumonia in Children" was published in 2024. Journal: Emerg Med Int.

# Clinical Features and Biomarkers for Early Prediction of Refractory Mycoplasma Pneumoniae Pneumonia in Children

**DOI:** 10.1155/2024/9328177

**Published:** 2024-01-05

**Authors:** Qin Chen, Tingting Hu, Ling Wu, Lumin Chen

**Affiliations:** ^1^Department of Respiratory Medicine, College of Clinical Medicine for Obstetrics & Gynecology and Pediatrics, Fujian Medical University, Fujian Children's Hospital (Fujian Branch of Shanghai Children's Medical Center), Fuzhou 350014, China; ^2^Department of Cardiology, College of Clinical Medicine for Obstetrics & Gynecology and Pediatrics, Fujian Medical University, Fujian Children's Hospital (Fujian Branch of Shanghai Children's Medical Center), Fuzhou 350014, China; ^3^Infectious Department, College of Clinical Medicine for Obstetrics & Gynecology and Pediatrics, Fujian Medical University, Fujian Children's Hospital (Fujian Branch of Shanghai Children's Medical Center), Fuzhou 350014, China

## Abstract

**Objective:**

The study aimed to analyze the clinical characteristics of children with RMPP and to explore the biomarkers for the early prediction of RMPP, thus providing references for the clinical diagnosis and treatment of RMPP in children.

**Methods:**

Baseline clinical characteristics, clinical symptoms, physical examination, chest imaging, and laboratory indicators between children with RMPP and general refractory mycoplasma pneumoniae pneumonia (GMPP) were compared. Multiple logistic regression analysis was used to determine independent risk factors for RMPP. ROC curves were adopted to analyze the predictive values of biomarkers.

**Results:**

The RMPP group had more severe clinical symptoms and manifestations on imaging (including pleural effusion, pulmonary consolidation, and pulmonary atelectasis), a higher incidence of extrapulmonary complications, and a longer duration of hospital stays. Results of multiple logistic regression analysis showed that serum D-dimer (OR = 8.169, *P* < 0.001), C-reactive protein (CRP) (OR = 1.146, *P* < 0.001), and lactate dehydrogenase (LDH) (OR = 1.025, *P* < 0.001) levels were independent risk factors for RMPP. The area under the receiver operating characteristic curve (AUROC) in RMPP prediction was 0.841, 0.870, and 0.893 for serum levels of D-dimer, CRP, and LDH, respectively (*P* < 0.001), with a cutoff value of 1.47 ng/ml, 39.34 mg/L, and 379 IU/L, respectively.

**Conclusions:**

Serum D-dimer, CRP, and LDH levels were related to the severity of mycoplasma pneumoniae pneumonia in children and had potential as biomarkers for the early prediction of RMPP, suggesting great applicative values for the early diagnosis and timely intervention of children with RMPP in clinical practice.

## 1. Introduction

Mycoplasma pneumoniae pneumonia (MPP) is a common disease of the respiratory system in children caused by mycoplasma pneumoniae (MP), with an incidence of approximately 10%–40% [1, 2]. MP is one of the most common causes of community-acquired pneumonia in children and adolescents. In recent years, the risk of MP infection has increased in the Chinese population. Epidemiological studies have shown that MPP has an epidemic outbreak every 3-4 years in European countries [3, 4]. More than 85% of MP strains among pediatric patients in China have been reported as macrolide-resistant MP, which can potentially cause severe and even extrapulmonary diseases. The global increase in macrolide-resistant MP is of concern due to limited therapeutic options [1]. Based on this fact, MPP is divided into refractory mycoplasma pneumoniae pneumonia (RMPP) and general mycoplasma pneumoniae pneumonia (GMPP) [5]. The prevalence of RMPP in children was 14.30%, with 6.83%, 20.86%, and 40.84% in those aged <4 years, 4–7 years, and ≥7 years, respectively [6].

The clinical presentation and manifestations of RMPP vary widely in different individuals and can affect all organs of the body. Children with RMPP may be complicated by pleural effusion, pulmonary atelectasis, gas accumulation in the mediastinum, pneumothorax, and necrotizing pneumonia. Some children with RMPP may develop respiratory distress, followed by rapid deterioration of their pulmonary functions, even requiring mechanical ventilation or extracorporeal lung support using extracorporeal membrane oxygenation (ECMO) [7], resulting in death. After conventional treatments, a recurrence of pulmonary lesions or a prolonged course of disease may still be observed, contributing to structural and/or functional lung abnormalities manifested by bronchiectasis [8]. In fact, these conditions are often associated with recurrent pulmonary infections in children and even exert a significant impact on pulmonary function in adults. To prevent progression and reduce relevant complications, early recognition and diagnosis are crucial for the appropriate treatment of RMPP in patients who are prone to clinical and radiological exacerbations during macrolide therapy. With the increase in the incidence and mortality of RMPP, the prevention of high-risk patients with RMPP has become a major concern in clinical practice [9, 10].

Currently, the diagnosis of RMPP has been challenging, with few significant features detected in laboratory or radiological evaluations, suggesting that there is no specific tool available for the diagnosis of RMPP [11]. Studies have shown that C-reactive protein (CRP), lactate dehydrogenase (LDH), erythrocyte sedimentation rate (ESR), percentage of neutrophils (NEPs), and the percentage of lymphocytes, together with the presence of dense solid pulmonary shadows, were significant predictors of RMPP [12–15]. Based on the above, this study was aimed to investigate clinical characteristics and explore biomarkers for early prediction of RMPP in children, providing references for the establishment of an efficient protocol for the early diagnosis of RMPP.

## 2. Materials and Methods

### 2.1. Study Design and Patients

This is a retrospective study. Children with MPP who were admitted to the Department of Respiratory Medicine, Fujian Children's Hospital, between January 2021 and December 2022 were enrolled. A flowchart of our research is detailed in Figure 1.

Inclusion criteria were the following: (1) patients aged 6 months-12 years; (2) patients who met the diagnostic criteria for MPP: positive results for the serologic test (positive IgM specific to MP, with IgM antibody titer >1 : 160) and nasopharyngeal secretions were positive for MP using polymerase chain reaction (PCR); and (3) patients who voluntarily underwent chest radiograph and/or CT examination.

Exclusion criteria were as follows: (1) patients with immunodeficiency diseases; (2) patients with respiratory diseases such as congenital bronchopulmonary dysplasia, pulmonary fibrosis, foreign bodies of the bronchial, asthma, tuberculosis, lung tumors, and noninfectious interstitial lung diseases; (3) patients with tumors, fracture trauma, tissue and organ fibrosis, and other diseases; and (4) patients with problems in specimen collection and incomplete data.

The study was approved by the Ethics Committee of Fujian Children's Hospital, Fujian Medical University. Patients were appropriately informed about treatment decisions. Informed consent was obtained from all patients.

### 2.2. Grouping of Patients

All patients were divided into 2 groups, including the GMPP group and the RMPP group. The diagnosis of RMPP was based on the presence of persistent fever (≥37.5°C) accompanied by clinical and radiological deterioration after azithromycin treatment for ≥7 days [9, 15]. Patients who met the diagnosis of RMPP were allocated into the GMPP group; others were classified into the GMPP group.

### 2.3. Data Collection

In the study, patient information was collected, including baseline clinical characteristics, laboratory results, and radiological findings. Baseline clinical characteristics, including age, sex, month and season of onset, hospital stay, clinical symptoms and signs, and extrapulmonary manifestations, were collected from both groups of children. Within 24 h of admission, all children were tested for respiratory pathogens and 2-3 ml of fasting venous blood was drawn for relevant laboratory tests, including MP-specific antibody titer tests, WBC count, percentage of NEP, CRP, LDH, procalcitonin (PCT), D-dimer, and tumor necrosis factor alpha (TNF-*α*). Imaging examinations mainly included chest radiographs and/or CT throughout the course of the disease, from which the extent of involvement, type of lesions, and intrapulmonary complications such as pulmonary atelectasis, pleural effusion, and pulmonary necrosis were collected.

### 2.4. Statistical Analysis

Statistical analysis was performed using SPSS 23.0. Continuous data with normal distribution were described with mean ± standard deviation (SD), and Student's *t*-test was used for comparison between the groups. Continuous data with a skewed distribution were presented with median and interquartile range (IQR), and the Mann–Whitney *U* test was used for comparison between the groups. Categorical data were expressed as frequency and percentage (%), and the chi-square test was used for comparison between the groups. Laboratory indicators of statistical significance in the comparisons were included as risk factors in the prediction of RMPP by using stepwise backward logistic regression. Receiver operating characteristic (ROC) curves were plotted, and the area under the curve (AUC) was calculated to evaluate the predictive value of laboratory indicators for RMPP. A two-sided *P* < 0.05 was considered as statistically significant.

## 3. Results

### 3.1. Comparison of Clinical Characteristics between the RMPP and GMPP Groups

In this study, 8 of 476 patients withdrew from the study. A total of 468 children with MPP were included finally, of which 156 (33.33%) were in the RMPP group and 312 were in the GMPP group.

As shown in Table 1, there were 55.77% males and 51.28% females in the RMPP group, with a mean age of 6.23 ± 2.89 years. RMPP occurs primarily in summer (36.54%) and in autumn (30.13%). However, there were no significant differences between the two groups in terms of sex, age, and season of onset (*P* > 0.05).

In terms of clinical symptoms, all patients in the RMPP group had fever, and the proportion of shortness of breath was significantly higher in the RMPP group than in the GMPP group (23.08% vs. 6.41%, *P* < 0.001); in contrast, the proportions of runny nose (36.90% vs. 8.50%, *P*=<0.001) and gastrointestinal symptoms (26.92% vs.18.59%, *P*=0.047) in the GMPP group were significantly higher than those in the RMPP group. However, the percentage of cough was as high as 94.87% in the RMPP group and 98.08% in the GMPP group, but their difference was not statistically significant (*P* > 0.05).

In terms of physical examination, the proportion of three concave signs (manifested as the suprasternal fossa, supraclavicular fossa, and concave intercostal space) was significantly higher in the RMPP group than in the GMPP group (10.90% vs. 2.56%, *P* < 0.001). The proportion of moist rales was 52.56% in the RMPP group and 46.79% in the GMPP group, but their difference was not statistically significant (*P* > 0.05).

In terms of pulmonary imaging, the proportions of pulmonary consolidation (79.49% vs. 41.99%, *P* < 0.001), pulmonary atelectasis (5.77% vs. 1.6%, *P*=0.013), and pleural effusion (30.77% vs. 2.24%, *P* < 0.001) in the RMPP group were all significantly higher than those in the GMPP group.

Furthermore, the proportion of extrapulmonary complications in the RMPP group was significantly higher than the GMPP group (37.18% vs. 16.99%, *P* < 0.001).

Extrapulmonary complications refer to the symptoms and signs of damage to other systems other than the respiratory system, including the digestive system, cardiovascular system, blood system, nervous system, urinary system, skin sores, and joint pain.

The mean duration of hospital days in the RMPP group was also significantly longer than that of the GMPP group (11.09 ± 4.25 vs. 8.27 ± 3.12, *P* < 0.001).

### 3.2. Comparison of Laboratory Indicators between the RMPP and GMPP Groups

As shown in Table 2, comparisons of laboratory indicators between the RMPP and GMPP groups showed that serum levels of CRP, LDH, PCT, and D-dimer were significantly higher in the RMPP group than in the GMPP group. However, the percentage of NEPs was significantly higher in the GMPP group than in the RMPP group. Differences in WBC count and TNF-*α* between the two groups were not statistically significant (*P* > 0.05).

### 3.3. Logistic Regression for Risk Factors of RMPP

Multiple logistic regression analysis showed that serum levels of D-dimer (OR = 8.169, *P* < 0.001), CRP (OR = 1.146, *P* < 0.001), and LDH (OR = 1.025, *P* < 0.001) were independent risk factors for RMPP. The linear probability model was as follows: logit (*P*) = −16.226 + 2.100*X*1 + 0.136*X*2 + 0.024*X*3 (Table 3).

### 3.4. Predictive Values of Serum D-Dimer, CRP, and LDH Levels for RMPP Using ROC Curves

To explore the predictive value of serum D-dimer, CRP, and LDH levels for RMPP, the ROC curves were plotted, and the AUC was calculated. The results showed good predictive values of serum D-dimer, CRP, and LDH levels for RMPP, with AUROC of 0.841, 0.870, and 0.893, respectively (Figure 2). The optimal cutoff point was determined according to the Youden index. Specifically, the optimal cutoff point of 1.47 ng/ml for the serum D-dimer level revealed a sensitivity of 64.74% and a specificity of 98.72% for the detection of RMPP, the optimal cutoff point of 39.34 mg/L for the serum CRP level revealed a sensitivity of 60.89% and a specificity of 94.55% for the detection of RMPP, and the optimal cutoff point of 379 IU/L for the serum LDH level revealed a sensitivity of 66.67% and a specificity of 93.91% for the detection of RMPP (Table 4).

## 4. Discussion

RMPP is usually characterized by a long course of disease, a poor therapeutic efficacy, and numerous complications that can even endanger the lives of children. The present study found that serum levels of D-dimer, CRP, and LDH were independent risk factors for RMPP, which laid a basis for early identification of RMPP and may be of great help in the diagnosis and prognosis of these children.

As reported, the most common clinical symptoms of RMPP were composed of cough (no sputum at the beginning and small to moderate bloodless sputum later), fever, chills, sore throat, headache, hoarseness, myalgia, and general malaise [16] and would worsen after 7 days of macrolide therapy, accompanied by persistent fever, pulmonary exacerbation in radiological findings, and extrapulmonary complications [17]. All of this was consistent with the clinical symptoms of children with RMPP observed in this study. Additionally, we also found that clinical symptoms were more severe in the RMPP group compared to the GMPP group, with fever observed in all children and a percentage of shortness of breath of up to 23.08% in the RMPP group. Furthermore, compared to those with GMPP, the images also presented with more severe manifestations in children with RMPP, with proportions of pulmonary consolidation, pulmonary atelectasis, and pleural effusion of 79.49%, 5.77%, and 30.77%, respectively.

In this study, 126 children (37.18%) with RMPP had extrapulmonary complications, which was significantly more than those in the GMPP group. Furthermore, the mean duration of hospital stays was 11.09 ± 4.25 in the RMPP group, which was also higher than the GMPP group with statistical significance. The abovementioned findings were in agreement with those reported in previous studies. Gong et al. [15] identified that persistent fever (>10 days), pleural effusion, extrapulmonary complications, pulmonary consolidation detected in chest radiography, and CRP > 40 mg/L could be used for early evaluation of RMPP by using a fixed-effects model or a random-effects model. In addition, Choi et al. [18] showed that respiratory distress, oxygen saturation <90%/cyanosis, oxygen support during hospitalization, lobar pneumonia on admission, and extrapulmonary complications were independent risk factors for RMPP, which was similar to the results of the present study.

The pathogenic mechanisms of RMPP are complex and include mainly direct pulmonary cell injury and immune response-induced injury. Currently, RMPP is considered to be related to airway mucus hypersecretion, hypercoagulable state, bacterial or viral infection, and excessive immune response due to the community-acquired respiratory distress syndrome (CARDS) toxin [19, 20]. Based on relevant basic research results and literature reports, this study selected 7 highly correlated biomarkers for the study of RMMP prediction indicators. CRP is one of the important indicators of inflammatory response [21], which has been widely used for assessing disease severity and treating inflammatory conditions. In addition, serum D-dimer levels have been recognized as a specific marker of the fibrinolytic system and an indicator of monitoring inflammations and severe infections [22]. The elevated level of D-dimer is possibly attributed to the injury of vascular endothelial cells caused by the excessive inflammatory response, which may be related to the mechanism of pulmonary injury in RMPP. Additionally, increased LDH activity has been found to be associated with pulmonary inflammation and hypoxia. High serum LDH levels showed the potential to predict an inadequate response to glucocorticoid treatment [23].

In this study, the results of multiple logistic regression analysis showed that serum D-dimer, CRP, and LDH levels were independent risk factors for RMPP; AUROCs for serum D-dimer, CRP, and LDH levels in the prediction of RMPP were all more than 0.8 (0.841, 0.870, and 0.893, respectively), suggesting their good predictive values in RMPP. Although the sensitivity of these cutoffs is lower than 65%, the specificity is higher than 93%, which can effectively exclude non-RMPP patients, thereby reducing the misdiagnosis rate. Similar to these findings, Zhang et al. also observed that the levels of CRP, LDH, and interleukin-6 (IL-6) were significantly higher in patients with RMPP than those with GMPP, indicating that they may be important predictors of RMPP in children and could facilitate the early identification of RMPP [21]. Meanwhile, the optimal cutoff points for serum D-dimer, CRP, and LDH levels for detecting RMPP were found to be 1.47 ng/ml, 39.34 mg/L, and 379 IU/L, respectively, which were comparable to the values of a case-control study (2.10 ng/ml, 343.08 mg/L, and 375 IU/L for serum levels of D-dimer, CRP, and LDH, respectively) [24]. Based on the abovementioned results, it could be inferred that serum levels of D-dimer, CRP, and LDH may have a certain value for clinical application.

There were several limitations in this study. First, as a single-center study, this study may have selection bias compared to multicenter studies. Second, a paired design was not performed and the patients in the RMPP group were not matched with those in the GMPP group for certain parameters, which may affect the statistical efficacy of the results. Finally, no joint prediction using multiple indicators was performed. Therefore, in the future, a multicenter-paired study should be conducted to further study the joint prediction of RMPP based on multiple indicators.

## 5. Conclusions

In conclusion, serum levels of D-dimer, CRP, and LDH are independent risk factors for RMPP and have high specific predictive values though low sensitivity for the early identification of RMPP. Early detection of RMPP within 24 hours of hospital admission may guide therapy revision for patients to reduce mortality.

## Figures and Tables

**Figure 1:** Flowchart of the study group.

**Figure 2:** ROC curves for D-dimer, CRP, and LDH for the prediction of RMPP.

**Table 1:** Comparison of clinical characteristics between the RMPP and GMPP groups (*n* = 468).

Factors	RMPP (*n* = 156)	GMPP (*n* = 312)	*t*/*χ*^2^	*P* value
*Sex*			0.840	0.359
Male	87 (55.77%)	160 (51.28%)		
Female	69 (44.23%)	152 (48.72%)		
*Age (years)*	6.23 ± 2.89	5.57 ± 3.02	2.294	0.218
*Onset season*			6.117	0.106
Spring	28 (17.95%)	32 (10.26%)		
Summer	57 (36.54%)	113 (36.22%)		
Fall	47 (30.13%)	111 (35.58%)		
Winter	24 (15.38%)	56 (17.95%)		
Clinical symptoms: fever	156 (100%)	249 (79.81%)	36.40	<0.001
Clinical symptoms: cough	148 (94.87%)	306 (98.08%)	3.682	0.055
Clinical symptoms: shortness of breath	36 (23.08%)	20 (6.41%)	27.424	<0.001
Clinical symptoms: runny nose	18 (8.50%)	115 (36.90%)	32.777	<0.001
Clinical symptoms: gastrointestinal symptoms	29 (18.59%)	84 (26.92%)	3.943	0.047
Physical examination: moist rale	82 (52.56%)	146 (46.79%)	1.386	0.239
Physical examination: three concave sign	17 (10.90%)	8 (2.56%)	14.283	<0.001
Lung imaging: lung consolidation	124 (79.49%)	131 (41.99%)	58.975	<0.001
Pulmonary imaging: atelectasis	9 (5.77%)	5 (1.6%)	6.222	0.013
Lung imaging: pleural effusion	48 (30.77%)	7 (2.24%)	81.599	<0.001
Extrapulmonary complications	58 (37.18%)	56 (16.99%)	20.874	<0.001
In hospital (day)	11.09 ± 4.25	8.27 ± 3.12	7.355	<0.001

**Table 2:** Comparison of laboratory indicators between the RMPP and GMPP groups (*n* = 468).

Index	RMPP (*n* = 156)	GMPP (*n* = 312)	*t*	*P* value
WBC (×10^9^/L)	7.76 ± 3.12	8.02 ± 4.52	−0.727	0.467
NEP (%)	58.69 ± 13.59	63.54 ± 14.07	−3.597	<0.001
CRP (mg/L)	42.13 ± 10.21	26.04 ± 9.15	17.233	<0.001
LDH (IU/L)	414.79 ± 72.76	292.98 ± 57.36	19.749	<0.001
PCT (ng/mL)	0.14 ± 0.09	0.11 ± 0.07	3.648	<0.001
D-dimer (ng/ml)	2.06 ± 1.08	0.83 ± 0.39	17.795	<0.001
TNF-*α*	3.19 ± 0.57	3.07 ± 0.42	1.557	0.120

**Table 3:** Logistic regression analysis for risk factors of RMPP.

Index	*B*	S.E	Wald *χ*^2^	*P*	Exp (B)	95% CI	
						Lower bound	Upper bound
D-dimer (*x*1)	2.100	0.374	31.595	<0.001	8.169	8.169	3.927
CRP (*x*2)	0.136	0.023	34.378	<0.001	1.146	1.146	1.095
LDH (*x*3)	0.024	0.004	39.565	<0.001	1.025	1.025	1.017

**Table 4:** Predictive values of serum D-dimer, CRP, and LDH levels for RMPP.

Index	Cut off value	Sensitivity (%)	Specificity (%)	AUC	Std. error	95% CI	*P* value
D-dimer	1.47	64.74	98.72	0.841	0.022	0.798–0.884	<0.001
CRP	39.34	60.89	94.55	0.870	0.017	0.837–0.903	<0.001
LDH	379.00	66.67	93.91	0.893	0.015	0.864–0.923	<0.001

## Data Availability

The data that support the findings of this study are available from the corresponding author upon request.
